# Design of an Interactive Two-Way Telemedicine Service System for Smart Home Care for the Elderly

This article has been retracted.

**DOI:** 10.1155/2021/6632865

**Published:** 2021-04-14

**Authors:** Fang Li

**Affiliations:** Jiangsu Vocational College of Medicine, Yancheng, Jiangsu 224005, China

## Abstract

In this paper, we deeply analyse and study the interactive telemedicine service system for elderly care in smart homes and design a data summarization method for large concurrent scenarios. The method first parses and reconstructs the data received by the system initially and then stores the reconstructed valid data into the local database, which realizes the fast data summarization under the heavy concurrency scenario. Secondly, a multiformat data adaptation method is designed for the problem that the data to be provided and processed are in various formats. The method uses a unified data format and adaptation process constraints to achieve centralized management of heterogeneous data from multiple sources, which provide a unified data support service for the system and upper-layer applications. Again, to deal with the application problem of highly correlated data, the data-sharing system provides data for each functional component of the telemedicine platform according to business requirements based on standardized data structure and unified storage management. This enables the barrier-free flow of multisource highly correlated data. When the consultation is in progress, the doctor can communicate with the patient with video and audio devices and, at the same time, can access the patient's historical medical records and the medical records uploaded by the patient; after the consultation is completed, the consultation doctor needs to fill in the consultation record. The consultation assistance module can statistically analyse the workload of doctors and other information according to the background data, and the telemedicine system will play an increasingly important role in the medical and health care business.

## 1. Introduction

The concept of telemedicine was first proposed by American scholars, which refers to the use of data technology, information technology, and communication technology as a basis to take advantage of the technical advantages of medical disciplines and advanced equipment resources of large general hospitals as well as specialized hospitals, in order to carry out the information system application of remote medical consultation and treatment, medical and health consultation, and precise collection of multisource heterogeneous data of various medical devices [1]. Data processing and network collaboration are the foundation of telemedicine [2]. Limited by the data processing and sharing capabilities and network bandwidth at that time, early telemedicine could only provide services in health consultation, medical consultation, and long-distance transmission of medical images [3]. With the continuous development of big data processing, cloud computing, and other emerging data technologies, telemedicine has developed a variety of telemedicine service modes such as teleconsultation, telecardiology, and telemedicine teaching [4]. With the development of data processing and sharing models, more medical service modalities will be developed and applied to social services [5]. Population aging is a product of economic and social development, and as an irreversible objective progress trend, it has become a major crisis faced by human society in the 21^st^ century [6]. With the development of related technologies and the gradual maturity of the industry, the design and development of senior care products have become abundant and diverse [7]. However, at present, the industry-standard coverage of senior products is not comprehensive; the positioning of products is not clear; the quality and safety of products are yet to be tested in the market, and the overall development status is not satisfactory [8]. Due to the special nature of the elderly group, the current acceptance of intelligent senior care products is generally low [9]. The main reason for this is that the functional positioning of the products does not match the urgent needs of the elderly, resulting in many intelligent senior care products being inconvenient to use and impractical in function, and the selling price is much higher than the consumption level of the elderly [10].

Rhoads and Rakes in a study of elderly care in Iceland found that formal care (skilled nursing facility or team) was chosen by elderly people who could not take care of themselves, while self-care elderly people chose more informal care, and informal care subjects must be considered in the elderly care system [11]. Macis et al. mentioned that the family care community model needs to be established, promoting the implementation of a long-term care insurance system (LTC) can effectively alleviate the problem of elderly people with disabilities [12]. Braley et al. pointed out that an important force in the provision of elderly care services is volunteer organizations, which play an active role in changing the concept of elderly care [13]. Costa et al. mentioned that the construction of a senior-friendly community should focus on several key factors, such as the paradigm of senior service provision, the degree of specialization of senior service, multicultural and recreational services, and the efficiency and duration of senior service, and the social work of the elderly should also pay attention to the disability and spiritual comfort of the elderly [14]. Stephens et al. mentioned that the main reasons that hinder the development of home-based services are insufficient funding and insufficient demand, and before its development is mature, it is still mainly provided by the government or governmental cooperative units, but home-based services can improve the quality of life of the elderly, enhance their sense of security, and also solve certain employment problems [15]. Chaet et al. analysed the interview data through semistructured interviews with elderly people at home and used phenomenological research methods to extract five urgent main service needs of elderly people at home for integrated medical care services, such as general medical treatment, health management, health education, Chinese medicine for the treatment of diseases, and personalized health and should actively promote graded medical treatment [16]. Fatta et al. mentioned that the path to realizing the “integrated medical and nursing care” health management service model mainly includes four aspects: concept advocacy, institutional guarantee, integration of existing medical structures and resources of elderly institutions, and talent training [17]. It is necessary to establish a hierarchical diagnosis and treatment system based on family doctors and establish a sound health management service industry and market supervision system for the elderly [18]. In her dissertation, Batsis talked about the government-led multiparty participation in the joint construction of a new elderly care service system suitable for China's social development needs, and the gradual construction of a new model based on the special and diversified demand characteristics of the elderly, with home care as the main focus, community care as a supplement, and institutional care as a guarantee [19] in combination with the actual development of the situation to broaden medical security, elderly care security, and focus on the emotional needs of the elderly, personalized elderly needs, and so forth [20].

To reasonably respond to the current situation of aging development and accelerate the integration of the Internet and elderly service industry, this paper starts from the integrated medical and nursing care elderly service model and analyses the current situation of elderly care and the research status of the elderly service model and elderly products. Through literature review, questionnaire research, directed interview, participatory observation, and experience, combined with qualitative research, the user needs under the integrated medical care model are summarized and analysed, and the methodological principles of the human-environment interaction model and interactive system model are selected as a guide to formulate a series of product design strategies and design principles under the integrated medical care model and carry out a series of product design planning layout, through product. The innovative design method is used to explore the needs of multiple target users and position the product functions to meet the needs of the service subjects and service objects for “medical care” functions under different usage scenarios. Through the design practice of the series of products, the functions of medical testing, health guidance, rehabilitation training, and multifunctional care are completed, and finally, the organic connection between the elderly and the medical care service personnel is realized through the intervention of innovative products to achieve the purpose of healthy aging. Finally, through design and practice, we provide the elderly, medical and nursing staff, and caregivers with products that meet the needs of the environment, such as health testing, elderly care, chronic disease management, and rehabilitation training, to better serve the application and promotion of the integrated medical and nursing care model.

## 2. Smart Home Interactive Two-Way Medical Service System Analysis and Design

### 2.1. Interactive System Design

Scholars have interpreted the home care service from different perspectives. Hsu points out that, as families tend to be smaller, the function of old-age care is weakening, and the average life expectancy of the elderly is increasing; people gradually prefer integrated social old-age care, which allows the elderly to enjoy help from various social parties while not being separated from their families of origin [21]. To meet all these needs, the home care service is proposed; the essence of which is that social organizations provide labour care services; families provide spiritual life care services, and the state collectively and individually share material life care services. Bearss et al. pointed out that the home care service is the provision of services related to the life, housekeeping, nursing care, and spirituality of the elderly, and it is a supplement and update of traditional old age [22]. Cardinale pointed out that the home care service is when the elderly live at home and social institutions come to their homes to provide day care or special care for the elderly [23]. In summary, home care service is a family-centred service that focuses on meeting the actual needs of the elderly without leaving the original living environment, relying on a service platform and providing a full range of services to the elderly in terms of living, housekeeping, medical care, health care, and spiritual cadetship through the integration of social resources. The services are provided in the form of day care centres, service stations, or direct home visits so that the elderly can enjoy services close to their homes, as shown in Figure 1.

The “Internet Home Senior Care” service is a new senior care service that combines Internet technology and related technology products based on home senior care service and uses Internet technology to fully mobilize and allocate the resources of the community and senior care institutions, to improve the level of home senior care service. Based on this new service, the elderly can order professional senior care services at home according to their needs. Not only that, the service provider is no longer limited to a small area, but the organization can accept a wide range of orders through the Internet platform, and one service provider may be able to cover the whole city. Not only can the Internet fully mobilize resources, but it can also enhance the professionalism of the services. For example, within a city, the Internet-based platform for senior care service providers has a massive overlap in the service areas of multiple agencies due to the expanded scope of services. For users, the selectivity of services is increased. Under the situation of benign competition, the senior care institutions continuously improve their service quality and specialization. At present, in the service of intelligent home care, the form of intelligent products is too single and the content tends to be homogenized, lacking innovative points. However, as the living standard of the elderly continues to improve, a single product form can no longer meet the diversified needs of its users. In this case, services with good experience can be a turning point in the field of aging in place. How to use the tools and methods of service design rationally to explore in-depth the needs of the elderly in the smart aging-in-place service and the needs of other relevant stakeholders (such as relatives, neighbours, community managers, service workers) and strive to improve the satisfaction of each stakeholder in the service system. Overall, the intervention of service design concept in the smart aging-in-place service can be considered from two perspectives: the perspective of system integration and the perspective of user experience, as shown in Figure 2.

Service design is a more systematic and holistic way of thinking. Smart aging in place involves multiple service scenarios and stakeholders, and by using the tools and methods of service design, it can help to provide systematic solutions to meet the needs of multiple parties in establishing services that focus on the experience of the elderly. Firstly, the needs of the elderly users are always the centre of the smart home care service system; at the same time, the needs and interests of the users at the whole service end are taken into account, mainly including relatives, friends, neighbours, community managers, service workers, whose interests are directly related to the quality of the elderly service. Secondly, we consider all aspects of senior care services from different perspectives. Thus, we can provide higher quality community senior care services and improve the service experience of the elderly. All designs in service design revolve around the needs of users, so the needs and experiences of elderly users and related stakeholders should be considered in smart aging-in-place services. Service providers need to recognize the diversity and hierarchy of the needs of the elderly, deeply understand the real needs of the elderly, and pay attention to the real scenarios of the elderly service usage. From the perspective of user experience, it is necessary not only to meet usability, ease of use, and efficiency at the functional level but also to evoke the psychology that elderly users want to use and are willing to participate in the service while receiving it.

### 2.2. Analysis of Smart Home Telemedicine Services

To better solve the data aggregation and data adaptation problems, this section is designed as a data gateway under the general framework of the data-sharing system. The essence of the data gateway is an encapsulated module that contains core functions related to data parsing and adaptation. The purpose of this design is to make the logical structure of each part of the system clearer and more importantly, to make the development of similar systems less difficult in the future. The data gateway is responsible for solving the problem of data interaction between the platform and external systems, and its interaction objects are the wearable devices supported by the platform and the business systems of medical examination organizations [24]. The main role is to collect and adapt the sports health data and medical checkup data from the above sources. According to the business requirements, the data gateway of the telemedicine platform is designed into three parts in terms of system structure, respectively: data parsing and classification framework, gateway local persistent storage framework, and data integration and upload framework. It realizes the functions from external device data aggregation, then to gateway local persistence, then to data uploading to platform unified storage, and finally to data distribution and invocation. The data gateway architecture is shown in Figure 3.

For medical examination report data, the data gateway deploys an FTP server to collect electronic medical examination report files. For the personal data from wearable devices of chronic disease tracking and management application (Love Care Heart) and sports and health application, the data gateway deploys socket-based data collection module and Restful Webservice based data collection module, respectively, according to the difference of communication protocols. At the same time, considering a large amount of data concurrency between the chronic disease tracking and management application and the sports health application, the data gateway deploys a database to store the collected raw data in real-time to prevent the blocking of the data adaptation process. The data gateway supports HTTP and TCP/IP based data transfer interfaces. Sports data and physical data are accessed to the gateway based on these interfaces. The gateway initially parses and reconstructs the incoming data and then provides feedback on the data analysis results. The valid data after a simple reconstruction of the original data is stored in the local database of the gateway. At the same time, the gateway will standardize and adapt the valid data in the local database and carry out unified storage of platform data. In this paper, to solve the problem of accessing multisource heterogeneous data for efficient standardization, this paper designs the method of initial parsing by the data gateway and then standardization. So, after combining the characteristics of each data such as medical examination reports, wearable devices, and cell phones, the main data structure is first designed as shown in Figure 3.

Teleconsultation medical system is mainly through the network mode to achieve the purpose of remote doctors to diagnose patients. In the process of diagnosing patients, doctors are no longer restricted by the time and location of the traditional medical service model and are completely free from the constraints of the hospital location and fixed working hours. A summary analysis of the survey data shows that teleconsultation has very strict requirements for the clarity of image acquisition and transmission, which means that the process of image acquisition cannot be inconsistent with the real objective phenomenon. At the same time, it is also necessary to ensure that the experts involved in the meeting can communicate and exchange with each other through the teleconsultation medical system and on this basis to ensure that the medical images and the patient's condition information can be transmitted in real time and closely linked to the hospital's information management system.

The main users involved in the teleconsultation system can be divided into different levels, and the operating authority of each level is also different. The main user levels are consultation centre, consultation hospital, specialist, administrator, and so on. Among the above users, the administrator is the core of the whole teleconsultation system, and his main role is to ensure the normal and smooth operation of the member system. In the process of a specific operation, he not only needs to manage the consultation centre efficiently but also needs to reasonably coordinate the work of patients, hospitals, and medical personnel, allocate reasonable time for system operation, reduce the pressure on the system, and ensure the normal operation of the system. The system needs to be coordinated with patients, hospitals, and medical staff, and the system needs to be operated at a reasonable time to reduce stress and ensure proper operation. The analysis of the system shows that patient-related data can be obtained from the system's user research canter, from the patient's online application for a consultation to the end of the doctor's diagnosis. Also, the data can be used and modified by the referrals, participating hospitals, and managers. When a patient uses the teleconsultation system, he or she first applies for the consultation qualification, and then the system administrator makes reasonable arrangements based on the actual situation of the consultation, and the specialist has to give the consultation result based on the consultation situation. During this process, the consultation specialist and the consultation administrator can send out data streams. Then, the consultation hospital will notify the patient to upload his basic information. From the above description, the top-level data flow delivery process of the teleconsultation system.

### 2.3. Systematic Evaluation Scheme Design

For the various terminals produced by different wearable device manufacturers and the different formats of terminal motion data and report data generated by 400 medical checkup institutions, a standardized adaptation method needs to be designed to standardize the collected data. This enables centralized storage of data to support the system and upper-layer applications, thereby improving the efficiency of data invocation for each application of the system and reducing resource usage [25]. This section introduces the design of the data adaptation process for wearable devices as an example. For the actual business scenario that requires comprehensive use through data from different sources, this section gives a method of invocation based on the results of the previous section. The convenient use of highly correlated data is realized. Taking the medical checkup application as an example, after the data is collected and adapted by the medical checkup application, multiple standardized data tables are invoked uniformly according to user requirements and forwarded directly to the data evaluation model module integrated with the telemedicine platform for calculation:

(1) $$\begin{array}{c} \phi \left(X,Y\right)=\left\{\begin{array}{c} \varphi \left(X\right)=X_{1},X_{2},\ldots ,X_{M},\\ \varphi \left(Y\right)=Y_{1},Y_{2},\ldots ,Y_{N}. \end{array}\right. \end{array}$$

In the appointment management module, the following operations are involved: patient condition information feedback, patient case data check, diagnosis result after patient consultation, advice, consultation application, consultation specialist list selection, consultation time determination, and so forth. Through the appointment management module, users can realize the functions of online consultation applications, accepting applications, reviewing applications, scheduling consultation, and notification of consultation information. The consultation management system can be divided into two basic modules: the consultation room management module and the video consultation management module. The consultation room management module is mainly responsible for arranging consultation rooms for users according to consultation applications and notifying patients and specialists to attend consultations according to consultation information promptly. The video consultation management module is mainly responsible for ensuring the smooth transmission of relevant data and information within the consultation room and creating a good environment for the communication of consultation experts. In the expert management module, users of the system can smoothly query all the expert information after successfully logging into the system, and some users with special authority can also update and maintain the expert information on time to ensure the authenticity and integrity of the expert information:

(2) $$\begin{array}{c} H=a_{1},a_{2},a_{3},\ldots ,a_{\left(m*n\right)}. \end{array}$$

In the consultation support management module, you can query the patient's historical medical records, track and manage the patient's condition, process the transfer application, query the evaluation information of the consultation specialists, and so forth:

(3) $$\begin{array}{c} \max\left(M,N\right)\geq K\geq M+N. \end{array}$$

In the process of teleconsultation, different participants can be selected to participate in the teleconsultation according to the actual situation, including users, experts, and managers. Next, the consultation centre module is used to build online web consultation rooms and adjust them to the actual situation. The consultation room management module contains more complex functions, including multipoint connection, video acquisition preparation, and screen synthesis. The second is the video consultation module. This module is mainly responsible for the acquisition and processing of audio information, video images, and so forth:

(4) $$\begin{array}{c} D\left(X,Y\right)=\sum_{k=1}^{K}\sum_{i=1}^{I}d_{k,i}\left(m,n\right). \end{array}$$

The patient's pathology is the information about the patient's condition, which is recorded and stored in the consultation system by the hospital to which the patient applies for teleconsultation so that the patient's condition can be viewed. The hospital to which the patient applies for teleconsultation stores the patient's medical history information in the hospital's management system in paper pathology or electronic form, in addition to the imaging information. The paper pathology, electronic pathology, and imaging information described above are all cases:

(5) $$\begin{array}{c} \text{VM}=\left\{\begin{array}{cc} \min & \frac{1}{2}{\left\|w\right\|}^{3}+C\sum_{i}\chi_{i}\delta_{i}\\ \text{s.t}. & y_{i}\left(w_{0}x_{i}+a\right)\leq 1-\chi , \end{array}\right.\\ A_{tsh}=\arccos\frac{{\left(P_{tsh}-Q_{tsh}\right)}_{i}^{2}\cdot {\left(P_{msh}-Q_{msh}\right)}_{i}^{2}}{\left(P_{tsh}-Q_{tsh}\right)\times \left(P_{msh}-Q_{msh}\right)},\\ A_{ksh}=\arctan\frac{\left(P_{ksh}-Q_{tsh}\right)\cdot \left(P_{ksh}-Q_{msh}\right)}{{\left(P_{ksh}+Q_{tsh}\right)}_{i}^{2}\times {\left(P_{msh}+Q_{msh}\right)}_{i}^{2}},\\ M=\left\{\begin{array}{c} w_{tsh}\times \frac{D_{shc}}{K_{shc}}+w_{msc}\cdot \frac{D_{shc}}{K_{shc}}=DT\;W,\\ w_{tsh}+w_{msc}=1. \end{array}\right. \end{array}$$

After the patient logs into the system, uploads his basic information into the system, and selects to save it, then the patient's information can be automatically stored in the system database, and the consultation centre will arrange the consultation time and place according to the patient's application requirements and inform the patient and the patient's chosen consultation specialist of the arrangement information promptly. Figure 3 reflects the contents of the consultation pathology filling page. The patient has to input basic information such as name, gender, age, the application number, and allergy history, into the system, and, after completing it, describe the patient's specific disease condition in as much detail as possible, and fill in the patient's phone number so that the patient can be contacted in time to arrange the consultation; meanwhile, the patient's related image cases and information should be uploaded into the system to prepare for the exhibition, as shown in Figure 4.

Contextual story design implies that the product is expressed based on a theme so that there is a story behind each product. It incorporates aesthetic sensitivity into the creative expression of the product so that a context can be created. When users see the products, they will have emotional resonance and can feel the context created by the product, thus evoking the user's subconscious touch and needs.

Emotional experience design can mobilize users' emotions. All emotional experiences are guided in two main directions: one is centred around changing users' negative emotions or guiding positive emotions, and the goal also represents the values of the emotional experience, for example, helping patients overcome their fear of hospitals or medical devices. Sometimes positive emotional guidance can also play a key role in motivating users to pursue long-term goals, for example, through clear and achievable goals and continuous feedback, so that users' positive emotions are constantly reinforced and they can work on their own to accomplish their goals, for example, using Ant Forest through the goal of “get a sapling” and the sapling's anthropomorphic feedback during the tree planting process. The anthropomorphic feedback reinforces users' emotions and internalizes them into personal goals, thus achieving them spontaneously. The second type is to increase user immersion experience, mainly applied in the game field, through different designs to convey different features in the game scenario and lead users to different emotions, through bold colours to promote the climax of the story and lead users to become happy, but also through low brightness colours and random layout to convey to users a “fragmented.” The plot atmosphere is also conveyed to users through low brightness colours and random layout. By conveying the emotion of the story to the user from the subconscious through some expressions, the user's emotion is constantly reinforced in the process of using the product.

## 3. Analysis of Results

### 3.1. System Performance Test Results Analysis

By understanding and analysing the actual work of the consultation system, we selected 10 functional points from the system that are frequently operated and have a large amount of data processing as the focus of this test. In the simulated test environment, the performance test tool was used to simulate users' load operations. The maximum number of concurrent users was set to 200, which was mainly used to record the average transaction response time of the system. The test results are shown in Figure 5.

The above results show that the response time of the 10 test items is within 4 seconds, and the response time of some items is even within 1 second, which meets the need of the system. Through the test, we can learn that the teleconsultation system can meet the design requirements, the functions can meet the requirements of actual teleconsultation, and the system data security is also guaranteed, which further promotes the development of China's telemedicine and plays a pivotal role in promoting the development of medical career. The functions available in the teleconsultation system are complete and match the design requirements. The administrator can efficiently manage the information of experts and patients through the system and meet the demand for real-time communication. The interface of teleconsultation is simple and friendly, which is more convenient for users and provides them with a good experience and meets their requirements for use. The security and confidentiality of the teleconsultation system are better, and the detection of user rights is better. The scope of operation of users with different rights is also different, which largely guarantees the security of the system, as shown in Figure 6.

The questionnaire data shows that the elderly have a higher demand for services such as remote viewing of health data, volunteers and health monitoring, and lower demand for psychological counselling and daily life. If the elderly are asked to purchase services at their own expense, the most popular choice is medical services, which according to Maslow's needs theory, is the most basic human need. For other services such as housekeeping and meal delivery, seniors think they can do these tasks by themselves and do not need to spend extra money to buy them. For mental health services, most seniors also think there is no need to spend on this area. The survey results show that seniors are more interested in volunteer services, smart health monitoring services, and remote viewing of health data services because these services are free or inexpensive. The above data show that the elderly in Baoding are not very enthusiastic about the purchase type of senior care services, which is not conducive to the progress and development of the senior care business, as shown in Figure 7.

The “Internet + home care” is a new senior care model with great potential, both technically and in terms of practical implementation; this model is an advanced method that has great significance and can play an important role. Of course, it has received a lot of attention, so our governmental departments have been actively issuing documents and advocating for its implementation in all regions since many years ago. However, it is clear from the research literature of each region that the development of most regions is very unpromising, and the most important problem is the imperfect management system. The contradiction between the imperfect system and the new model directly leads to the actual construction situation seriously deviating from the expected goal of the program. In the test results of this scenario, it can be seen from Figure 7 of the test results that the transaction processing speed reaches 39.195 transactions/second with 600VU concurrency, and the processing speed of failed transactions is 0.183 transactions/second, accounting for 0.46%, which is less than 5% of the requirement. Firstly, the implementation effect demonstrated from the perspective of the telemedicine system application and the data parsing, adaptation, and invocation functions of the data-sharing system were proved to be normal through actual usage scenarios. The performance of the system was then tested by tools, and the performance of the data gateway and database interface was directly verified to meet the design requirements through pressure testing. The research results of this paper were demonstrated by these two aspects. Given the high correlation of data required by telemedicine applications, this paper designs an application method to provide highly correlated data for each functional component of the telemedicine platform according to business requirements. Thus, the barrier-free flow of highly correlated data from multiple sources is realized.

### 3.2. Analysis of Application Results

After the system development work is finished, before the system is officially used, the major functional modules inside the system need to be tested to ensure that the whole system can operate normally and the functions that the system has can meet the needs of the users. It is a test of the whole system, considering the hardware, software, and operators, to check whether it has any nonconformity with the system specification. This kind of testing can find errors in the analysis and design of the system. For example, security testing is to test whether the security measures are perfect and can ensure that the system is protected from illegal intrusion. For example, stress testing is to test whether the system works properly under normal data volume as well as an overload (e.g., multiple users accessing at the same time). Based on the system requirement analysis, a test plan for the teleconsultation system was developed, with a network bandwidth of at least 100MLAN, using a Cisco switch to connect users to the system centre, and being able to provide a good network environment to guarantee real-time data transmission. The main reflection is the network topology composition of the teleconsultation system. The calculation process is shown in Figure 8.

The testing of the teleconsultation system mainly includes whether there is any abnormality in the account login; whether the system can detect the illegal account access to the system and give an alert; whether the account access authority meets the design requirements; whether the system functions are consistent with the design requirements; whether the system can operate according to the system design requirements; and so forth. In the process of testing the system, it is also necessary to test some special information to ensure that the system can operate according to the design requirements, in addition to testing the existing functions of the system. After all the test contents meet the requirements, the system can be handed over to the users. Test requirements: the user can successfully log into the system and can perform the corresponding operations according to the different permissions, and the system will detect and prompt for empty accounts.  Figure 9 shows the user login interface. Operation process: in the process of logging in, the user detects illegal input according to the different permissions of different users and observes whether it will affect the normal operation of the system. Detection results: in the process of login, if the user is illegal input, the system will prompt an illegal user name; if no password is entered or the password is wrong, then the system will prompt the wrong password; if the user is legal and the password is normal, the user can successfully login to the main page of the system and the page is displayed normally. Conclusion summary: if an illegal user tries to log into the system, the user name will be prompted as illegal; if the password is empty or wrong, the password will be prompted as wrong; if both the user name and password meet the requirements, then the user will be able to enter the login screen smoothly. Because user requirements will change appropriately, new user requirements should be accepted before the official operation. Therefore, in the testing session, appropriate adjustments should be made according to the latest requirements. In many system logins interfaces, to prevent violent cracking and other means, the form of verification code is usually added to cope with the situation. After communication with various parties, the 4-bit random verification code verification mode is added to the login window.

Using the proposed design principles and methods, we conducted a practical study of product design for elderly users using smart TVs as an example, validated the theory and method system through design practice, and further explored and practiced ways to improve the perception of elderly users in the design method. Based on the user-centered approach and principles of the methodology, focus groups were used to obtain and analyse the needs of elderly users in detail, and on this basis, the functional, cosmetic, and interactive interfaces were designed with corresponding target solutions. The results showed that the objective performance of the prototype was significantly better than that of the existing product and shortened the performance gap between novice and skilled users, and the overall subjective satisfaction of the design solution was also higher than that of the existing product, which fully verified the effectiveness and applicability of the product design method proposed in this paper, as shown in Figure 10.

The teleconsultation database holds a large amount of information and data and the main source of information in hospitals of different sizes and in different regions. The total amount of data and information is relatively large and contains a variety of data, so in the process of designing this system, the data is not stored on the server, but on the client-side. The specialists need to transfer the required information from the client to the server before the consultation is carried out, and the server can receive the information automatically.

## 4. Conclusions

To solve the problem of frequent and concurrent data generation for the system, this paper designs a method to collect data in a large concurrent scenario where the system first stores the valid data in the local database after the initial parsing and reconstruction of the received data and then performs standardized adaptation when integrating and uploading. Stability and efficiency of data collection are achieved to solve the problem of receiving data in a wide variety of formats, which in turn cannot effectively achieve efficient data sharing. The article designs a multiformat data adaptation method according to the unique characteristics of data. The method defines a unified data format and adaptation process to standardize data formats entering the telemedicine platform. Given the high correlation of data required by telemedicine applications, this article designs an application method to provide highly correlated data for each functional component of the telemedicine platform according to business requirements. Thus, the barrier-free flow of highly correlated data from multiple sources is realized. Thus, a feasible teleconsultation system is constructed, which uses a consultation centre model based on the consultation centre model and incorporates hospital consultation operations, and users have an obligation to register and enroll in the consultation centre before they can use the system. The main advantage of the teleconsultation system is that the whole system has a very clear and good structure and a high degree of purposeful concentration, which can further improve the efficiency of consultation.

## Figures and Tables

**Figure 1:** Interactive service design.

**Figure 2:** Methodology and steps.

**Figure 3:** Data gateway system architecture.

**Figure 4:** Schematic diagram of platform data interaction.

**Figure 5:** Test statistics.

**Figure 6:** Types of personal service needs of the elderly.

**Figure 7:** VUser-TPS.

**Figure 8:** Cross-validation results at different k values.

**Figure 9:** Three-dimensional plot of cross-validation accuracy.

**Figure 10:** Nursing care training score line graph.

## Data Availability

Data sharing not applicable to this article as no datasets were generated or analysed during the current study.
